The article "Iron application improves yield, economic returns and grain-Fe concentration of mungbean" was retracted in 2022. Reasons: compromised peer review; a conflict of interest; concerns about the authorship.

# Iron application improves yield, economic returns and grain-Fe concentration of mungbean

**DOI:** 10.1371/journal.pone.0230720

**Published:** 2020-03-27

**Authors:** Abdul Majeed, Waqas Ahmed Minhas, Noman Mehboob, Shahid Farooq, Mubshar Hussain, Sardar Alam, Muhammad Shahid Rizwan

**Affiliations:** 1 Department of Agronomy, Bahauddin Zakariya University, Multan, Pakistan; 2 Department of Plant Protection, Harran University, Sanliurfa, Turkey; 3 Department of Agronomy, Faculty of Agricultural Sciences, Ghazi University, Dera Ghazi Khan, Pakistan; 4 School of Veterinary and Life Sciences, Murdoch University, Murdoch, WA, Australia; 5 Department of Agronomy, University of Agriculture, Faisalabad, Pakistan; 6 Cholistan Institute of Desert Studies, The Islamia University of Bahawalpur, Bahawalpur, Pakistan; Omer Halisdemir Universitesi, TURKEY

## Abstract

Malnutrition is among the biggest threats being faced globally, and Pakistan is among the countries having high malnutrition rate. Pulses grown in Pakistan have lower amounts of micronutrients, especially iron (Fe) in grains compared to developed world. Biofortification, -a process of integrating nutrients into food crops-, provides a sustainable and economic way of increasing minerals/micronutrients’ concentration in staple crops. Mungbean fulfills protein needs of large portion of Pakistani population; however, low Fe concentration in grains do not provide sufficient Fe. Therefore, current study was conducted to infer the impact of different Fe levels and application methods on yield, economic returns and grain-Fe concentration of mungbean. Mungbean was sown under four levels of Fe, i.e., 0, 5, 10 and 15 kg Fe ha^-1^ applied by three methods, i) as basal application (whole at sowing), ii) side dressing (whole at 1^st^ irrigation) and iii) 50% as basal application + 50% side dressing (regarded as split application). Iron levels and application methods significantly influenced the allometry, yield, economic returns and grain-Fe concentration of mungbean. Split application of 15 kg Fe ha^-1^ had the highest yield, economic returns and grain-Fe concentration compared to the rest of Fe levels and application methods. Moreover, split application of 15 kg Fe ha^-1^ proved a quick method to improve the grain-Fe concentration and bioavailability, which will ultimately solve the Fe malnutrition problem of mungbean-consuming population in Pakistan. In conclusion, split application of Fe at 15 kg ha^-1^ seemed a viable technique to enhance yield, economic returns, grain-Fe concentration and bioavailability of mungbean.

## Introduction

Malnutrition is an important nutritional disorder that refers to the deficiency of basic nutrients in human diet. Malnutrition is grouped in two different categories, i.e., protein/energy malnutrition and micronutrient malnutrition [1]. Micronutrient malnutrition or “hidden hunger” occurs due to the deficiency of micronutrients in daily diet and half of the global population suffers from micronutrient malnutrition [2]. The lack of calories and proteins is the reason of protein/energy malnutrition, which is the most lethal type and 925 million people were affected by it during 2010 [3]. Women and pre-school children are the most vulnerable and at least 5 million children die every year as a result of micronutrient malnutrition [4]. Micronutrients such as zinc (Zn), boron (B) and Fe are required in small amount and their deficiency results in retarded growth and development in humans.

Iron is highly important for growth and development of immune system [5]. It also plays a role in photosystems [6]. Globally, Fe-deficiency is the most prevalent micronutrient disorder. Fe-deficiency causes high mortality rate, problems in pregnancy, low mental development and physical health and less productivity of work in adults [7]. Fe-deficiency affects oxygen supply and causes tiredness, decrease in immunity level and increases risk of blood anemia [8]. The recommended dietary allowance (RDA) of Fe for adult women is approximately 60 and 20 mg/day with low and high iron bioavailability diet, respectively [9]. In South Asia, approximately 88% of pregnant women and 63% of children between 5 and 14 years suffer from anemia [3, 10].

Pulses offer environmental and nutritional benefits; therefore, recommended in sustainable diets [11]. Moreover, Food and Agriculture Organization of the United Nations (FAO) recommend pulses as staple foods to fulfill the basic protein and energy requirements of the human diet [12]. Pulses are an excellent and cheap source of amino acids like glutamic acid, aspartic acid, lucien, isoleucine and phenylalanine [13]. Pulses also increase soil fertility due to its biological nitrogen fixation properties.

The per capita consumption of pulses in Pakistan is 16 g day^−1^ [14], and pulses provide approximately 25% of all Fe in the diet. Mungbean (*Vigna radiata* (L.) R. Wilczek var. *radiata*) is one of the important pulse crops consumed in the country [14–16], and has efficient digestibility than other pulses [17]. It has high nutritional value and readily available source of protein as it contains carbohydrate (51%), protein (24–26%), minerals (4%) and vitamins (3%). Pakistan was the second largest producer of mungbean in South Asia during 2009–10. Mungbean accounted for 16% of total pulses consumed in the country during 2009–10 [18].

Research on the nutritive value of mungbean has reported significant variations regarding Fe concentration in different genotypes [19]. Allen et al. [20] concluded that Fe, vitamin A and iodine are commonly deficient in mungbean and cause malnutrition. Therefore, increasing Fe concentration through breeding and agronomic techniques could solve the problem of malnutrition.

Biofortification is a promising, cost-effective, and sustainable technique of delivering micronutrients to a population that has limited access to diverse diets and other micronutrient interventions. Biofortification is a process of increasing the concentration of required mineral in staple crop through special means, including plant breeding and agronomical practices [21]. Petry et al. [22] suggested that biofortification is only sustainable and cheap agriculture-based technique to sort out the problem of Fe deficiency. Agronomic biofortification of micronutrients like Fe and Zn is considered as most appropriate and cheap method to cope this problem [23]. Agronomic biofortification considered as a short-term solution to increase the concentration of micronutrient but as compared to breeding it is easier and feasible to attain [24, 25]. Agronomic biofortification may offer a rapid solution to mineral deficiencies and represents a complementary approach to ongoing breeding programs [26].

Mungbean is highly nutritive and a cheap source of protein, carbohydrate and vitamins; however, low amount of Fe in its grains leads to malnutrition of the population dependent on it for Fe intake. Several studies around the world have evaluated the impacts of supplemental Fe application on growth and mineral concentration of mungbean; however, no studies have been conducted in Pakistan. Therefore, this study was conducted to infer the impacts of different Fe doses and application methods on growth, yield and grain-Fe concentration of mungbean. It was hypothesized that grain Fe content will linearly increase with increasing Fe dose. Moreover, different application methods will differ in their efficacy for Fe utilization and storage in grains.

## Materials and methods

This field study was conducted at Agronomic Research area, Bahauddin Zakariya University, Multan, Pakistan during spring season, 2017. Three soil samples (0–20 cm depth) were collected from different locations of the experimental soil before sowing to evaluate the fertility status of the experimental field. The soil was clay-loam with pH 8.30, soil organic matter content 0.98%, EC 1.74 dS m^-1^, available nitrogen (N) 0.023%, available potassium (K) 122 mg kg^-1^, available phosphorous (P) 6.00 mg kg^-1^ and available iron (Fe) 4.02 mg kg^-1^. Weather data during the whole experimental period was recorded and presented in Table 1.

**Table 1:** Weather data of experimental site during the whole course of experiment.

Months	Mean monthly temperature (°C)	Mean monthly relative humidity (%)	Total monthly rainfall (mm)
March	21.8	68.4	0.0
April	30.0	53.5	5.3
May	34.0	63.1	0.1
June	33.1	74.9	45.6

Source: Pakistan Central Cotton Committee (PCCC), Multan, Pakistan

### Experimental details

Seeds of mungbean variety Azri-2006 were collected from Arid Zone Research Institute (AZRI), Bhakhar, Pakistan. The experiment consisted of four Fe levels, i.e., 0 (regarded as control), 5 (regarded as low dose), 10 (regarded as medium dose) and 15 (regarded as high dose) Kg ha^-1^, whereas FeSO_4_ was used as Fe source. Three different application methods i.e., i) whole Fe as basal application as band placement (regarded as basal application), ii) whole Fe as side dressing with 1^st^ irrigation (regarded as side dressing) and iii) 50% of Fe as basal application and 50% as side dressing (regarded as split application) were used. Experiment was laid out in randomized complete block design under factorial arrangement. The application methods were considered as main factor, whereas Fe levels were regarded as sub factor. Experiment was replicated four times using net plot size of 1.5 m × 5 m.

### Crop husbandry

About 10-cm pre-sowing irrigation was applied before seedbed preparation. Seedbed was prepared by applying three cultivations with tractor-mounted cultivator followed by planking. The crop was sown on March 21, 2017 in 30 cm spaced rows using seed rate of 10 kg ha^-1^. Sowing was done by manually operated single row drill. Thinning was done at 2-leaf stage to maintain plant × plant distance of 10 cm. Fertilizers were applied at the rate of 23 kg and 55 ha^-1^ nitrogen (N) and phosphorus (P) using urea (46% N) and di-ammonium phosphate (18% N and 46% P_2_O_5_), respectively as sources. The whole amounts of N and P were applied at sowing in all application methods for uniformity. Hand hoeing was done to manage the emerging weeds. Four irrigations were applied to avoid moisture stress and last irrigation was applied before two weeks of harvest. Lufenuron (50 g L^-1^) was applied at the rate of 500 mL ha^-1^ to keep the crop free from army worms attack. The mature crop was harvest on July 07, 2017.

### Crop allometry

Four plants from each experimental unit were randomly selected to measure chlorophyll density. Chlorophyll density was measured by SPAD meter (Minolta Chlorophyll Meter SPAD-502DL). Leaf area was measured by destructive method using leaf area meter (DT Area meter, Model MK2, Delta T Devices, Cambridge, UK). All plants in 0.5 m row were harvested and their leaf area was measured. First data were recorded at 30 days after sowing (DAS) and 2^nd^ data were recorded at 50 DAS. The LAI was calculated by the equation suggested by Watson [27].

$$\mathrm{LAI}=\frac{\mathrm{Leaf}\;\mathrm{area}}{\mathrm{Land}\;\mathrm{area}}$$

Four plants were randomly selected from each experimental unit to measure crop growth rate (CGR). The plants were harvested, weighed fresh, brought to the laboratory and dried at 70°C in oven for 72 hours. The dried samples were weighed with the help of measuring scale. First sampling was done 30 DAS, whereas the second sampling was done at 50 DAS. The dry weight of plants was converted to dry weight m^-2^. The CGR was then calculated by the formula suggested by Hunt [28],

$$\mathrm{CGR}=\frac{W_{2}‐W_{1}}{t_{2}‐t_{1}}$$

Here, W_2_ = dry weight at 2^nd^ harvest, W_1_ = dry weight at first harvest, t_2_ = time at 2^nd^ harvest and t_1_ = time at 1^st^ harvest.

### Morphological and yield related traits

Ten randomly selected plants in each plot were used to record average plant height, number of sympodial and reproductive branches per plant. Average pod length and number of pods per plant was counted from these selected plants. Twenty randomly selected pods were used to record number of seeds per pod. All plants present in all experimental units were harvested at maturity. The harvested plants were sun dried for three days, tied into bundles and weighed using spring balance to record biological yield. After sun drying, all pods were separated, manually threshed and grains were weighed to record grain yield/experimental unit for each experimental unit, separately. Then grain and biological yields were converted into t ha^-1^ using unitary method. Three random samples of 1000 grains were taken from the seed lot of each experimental unit, weighed and averaged to record the 1000-grain weight. The harvest index was measured as the ratio of grain yield to the biological yield, expressed in percentage.

### Statistical analysis

Collected data were analyzed by Fisher’s Analysis of Variance (ANOVA) technique. Normality in the data was tested by Shapiro-Wilk normality test prior to ANOVA. The data were normally distributed; therefore, the analyses were executed on original data. Two-way ANOVA was used to test the significance in the data. The means were then separated by least significant difference test at 5% probability level where ANOVA indicated significant differences [29].

### Economic analysis

Economic analysis was conducted to assess the economic feasibility of different Fe levels and application methods. Fixed costs included land rent, seedbed preparation, seeds, fertilizers, plant protection measures and harvesting etc., whereas the variable cost included price of Fe fertilizer and labor charges incurred on application methods. Total income was computed based on existing prices of mungbean. Net income was computed by subtracting the total expenditure from gross income. Finally, benefit cost ratio was computed by dividing net income with total expenditure.

## Results

Different iron (Fe) levels, application methods and their interaction significantly altered crop growth rate (CGR) and leaf area index (LAI) (Table 2). However, number of roots/plant and chlorophyll density was significantly affected only by Fe levels and application methods, respectively (Table 2).

**Table 2:** Statistical summary of growth yield and related traits, grain-Fe concentration and economics of mungbean grown under varying iron levels and application methods.

Crop variables	Iron levels (Fe)	Iron application methods (M)	Fe × M
Number of roots/plant	*	NS	NS
Chlorophyll density (SPAD value)	NS	**	NS
Leaf area index	**	**	**
Crop growth rate (g m^-2^ day^-1^)	**	**	**
Number of monopodial branches/plant	**	**	**
Number of sympodial branches/plant	**	NS	**
Number of grains per pod	**	**	**
1000-grain weight (g)	**	**	**
Grain yield (t ha^-1^)	**	**	**
Biological yield (t ha^-1^)	**	**	**
Gross income (US$ ha^-1^)	**	**	**
Net income (US$ ha^-1^)	**	**	**
Benefit: cost ratio	**	**	**

* = Significant at p 0.05

** = Significant at p 0.01; NS = Non-significant

Split application with high Fe level had the highest LAI and CGR, whereas the lowest values of these traits were recorded in control treatment (Fig 1A and 1B). Similarly, split application of high Fe level had the highest number of lateral roots and chlorophyll density, whereas the lowest values were recorded for control treatment (Fig 1C and 1D).

**Fig 1:** Effect of different iron levels and application methods on leaf area index (A), crop growth rate (B), number of roots/ plant (C) and chlorophyll density (D) of mungbean ± SE (n = 4) Here B = Basal application of Fe; S = Side dressing of Fe; Chl = Chlorophyll; CGR = Crop growth rate.

Different Fe levels, application methods and their interaction significantly affected number of monopodial branches and sympodial branches, number of pods per plant, and number of grains per pod except the non-significant effect of application methods on number of sympodial branches/plant (Table 2). Split application with higher Fe dose observed the highest number of monopodial branches, sympodial branches, pods per plant, and number of seeds per pod of mungbean (Fig 2A–2D). The lowest number of monopodial branches, sympodial branches, pods per plant and seeds per plant were recorded from control treatment (Fig 2A–2D).

**Fig 2:** Effect of different iron levels and application methods on number of monopodial branches (A), sympodial branches (B) and pods per plant (C), and number of seeds per pod (D) mungbean ± SE (n = 4) Here B = Basal application of Fe; S = Side dressing of Fe.

Moreover, different Fe levels, application methods and their interaction had significant effect on 1000-grain weight, grain and biological yields, and grain-Fe concentration (Table 2). Split application of Fe at higher level observed the highest 1000-grain weight, grains and biological yields and grain-Fe concentration of mungbean (Fig 3A–3D). The lowest 1000-grain weight, grains and biological yields and grain-Fe concentration of mungbean were recorded from control treatment (Fig 3A–3D).

**Fig 3:** Effect of different iron levels and application methods on 1000-grain weight (A), grain yield (B), biological yield (C), grain-Fe concentration (D) mungbean ± SE (n = 4) Here B = Basal application of Fe; S = Side dressing of Fe.

Different Fe levels, application method and their interaction significantly affected the net income and BCR (benefit cost ratio) (Table 2). Higher dose of Fe achieve maximum returns in producing maximum gross income and BCR as compare to control where no Fe was applied. Maximum gross income and BCR were achieved by spilt application method with high Fe application. The lowest income and BCR ratio was recorded where no Fe was applied (Table 3).

**Table 3:** Economic analysis growing mungbean under different Fe levels and application methods.

Treatments		Total cost (US$ ha^-1^)	Gross income (US$ ha^-1^)	Net income (US$ ha^-1^)	Benefit: cost ratio
Application methods	Iron levels (kg ha^-1^)				
Control (No iron application)		463	1502 f	1039 f	3.20 f
Basal application	5	469	1552 de	1083 de	3.31 de
	10	471	1585 bc	1114 b-d	3.36 b-d
	15	473	1567cd	1094 c-e	3.31 c-e
Side dressing	5	469	1552 de	1083 de	3.31 de
	10	471	1591 bc	1120 bc	3.38 bc
	15	473	1606 b	1133 b	3.39 b
Split application	5	471	1575 b-d	1104 b-d	3.35 b-d
	10	472	1576 b-d	1194 b-d	3.33 b-e
	15	474	1668 a	1116 a	3.52 a

Means not sharing the similar letters, within a column, differ significantly from each other at p ≤ 0.05

## Discussion

The results indicated that high Fe level and split application had significant effect on number of roots per plant LAI, CGR and chlorophyll density (Fig 1A–1D). Split application of 15 kg Fe ha^-1^ produced higher number of roots per plant, as compared to rest of the Fe levels. The results indicated that Fe application resulted in better root proliferation that helped the plants to produce more number of roots (Fig 1C). Higher numbers of roots help the plants to access more nutrients and water [30]. High water availability at vegetative stage helps plant to maintain cell turgidity. Turgid cells increase the leaf size to harvest more light. Leaves play a major role in development of plant as they harvest sunlight, convert it into chlorophyll and store it for plant development. Moreover, leaves are a major source which transfer assimilates to seed or sink. The LAI of mungbean was increased with increasing Fe level (Fig 1). Fe plays a major role in enzyme activation because it is part of many enzymes, cytochrome which is involved in electron transport chain; synthesize chlorophyll and structure of chloroplasts [31]. The increase in leaf area enables plants to harvest more sunlight, which results in increased chlorophyll density, LAI and grain yield [32].

Micronutrients, especially Fe, play an important role in chlorophyll and enzymatic activity, which had great importance in photosynthesis and respiration [33]. Fe has greater role in process of photosynthesis and respiration [34]. It is reported that Fe has significant effect on the synthesis of growth regulators and in chlorophyll synthesis [35]. When leaves contain high chlorophyll content they appear lush green color with more size and weight. As the results shows that split application of 15 kg ha^-1^ Fe increased LAI, which intercept more light essential for plant metabolism.

Yield and nutritive value of seed are improved when plant completes its lifecycle under benign environmental conditions resulting in better performance at early stages. Results revealed that split application of 15 kg ha^-1^ Fe significantly affected agronomic and yield related traits and produced more grain and biological yield compared to control (Figs 2 and 3). The mungbean yield improvement directly depends on crop allometric traits i.e., LAI, number of pods per plant, pods length, number of seeds per pod and biological yield.

Application of Fe improves plant height of *Vigna radiata* and *Nigella sativa* [36]. Thus, higher plant height reveals more biomass production. Ziaeian and Malakouti [37] reported that Fe, Zn, Cu and Mn increased 1000-grain weight, grain yield, number of grains per spikelet and straw yield in wheat and also showed that Fe application had significantly increased the Fe content in grain. Our results also indicated that split application of 15 kg ha^-1^ Fe improved Fe content of mungbean seed. The reason behind high Fe content in seed is the continuous availability of Fe to mungbean plants throughout lifecycle. It was previously observed that Fe content of wheat improved by 21% by Fe application [38]. Similarly, Fe application also improved the Fe content in groundnut [39].

Iron application in staple crops such as in wheat improves benefit cost ratio [40]. Results indicated that iron level and split application had significant effect on benefit cost ratio (Table 3).

The field scale adaptability of any novel and emerging technique depends upon its economic feasibility. The economic analysis indicated that split application of 15 kg Fe ha^-1^ generated higher income and BCR compared to the rest of the Fe levels. Thus, 15 kg Fe ha^-1^ could effectively be used to improve the economic returns of mungbean (Table 3).

The overall objective of the current study was to improve the Fe concentration of mungbean grains through biofortification. The Fe application significantly improved the Fe concentration; thus, grains must be biofortified with Fe to improve the diet quality of the residents of the country. Nonetheless, Fe biofortification proved as an effective technique to solve the problem of Fe malnutrition in the country.

## Conclusions

The data on allometric, yield related traits, Fe concentration in grains and economic analysis revealed that split application of 15 kg ha^-1^ Fe produced higher yield, generated the highest income and improved grain Fe concentration. Therefore, split application of 15 kg ha^-1^ Fe is recommended for improving the yield, Fe concentration and productivity of mungbean in Pakistan as well as other parts of the world to solve the problem of Fe malnutrition. Nonetheless, higher Fe doses must also be tested for their possible effects on productivity and Fe concentration of mungbean.
